RETRACTED

# Analysis of Body Behavior Characteristics after Sports Training Based on Convolution Neural Network

**DOI:** 10.1155/2021/7006541

**Published:** 2021-07-20

**Authors:** Xinliang Zhou, Shantian Wen

**Affiliations:** ^1^School of Physical Education, Xihua University, Chengdu, Sichuan 610039, China; ^2^School of Physical Education, Huzhou University, Huzhou, Zhejiang 313000, China

## Abstract

The use of artificial intelligence technology to analyze human behavior is one of the key research topics in the world. In order to detect and analyze the characteristics of human body behavior after training, a detection model combined with a convolutional neural network (CNN) is proposed. Firstly, the human skeleton suggestion model is established to analyze the driving mode of the human body in motion. Secondly, the number of layers and neurons in CNN are set according to the skeleton feature map. Then, the output information is classified according to the fatigue degree according to the body state after exercise. Finally, the training and performance test of the model are carried out, and the effect of the body behavior feature detection model in use is analyzed. The results show that the CNN designed in the study shows high accuracy and low loss rate in training and testing and also has high accuracy in the practical application of fatigue degree recognition after human training. According to the subjective evaluation of volunteers, the overall average evaluation is more than 9 points. The above results show that the designed convolution neural network-based detection model of body behavior characteristics after training has good performance and is feasible and practical, which has guiding significance for the design of sports training and training schemes.

## 1. Introduction

Body behavior is one of the main characteristics in the process of human activity. With the development of science and technology, the research on human behavior has attracted a lot of researchers' attention worldwide. The current research methods mainly include attitude perception and action recognition [1]. Nakandala et al. [2] proposed a sensor-based behavior recognition system based on a deep recursive neural network (RNN), which integrates data from ECG, accelerometer, magnetometer, and other individual sensors to identify human behavior. Zhang and Ling [3] designed the structure and joint motion feature extraction of the two-channel deep convolution neural network model and extracted joint motion information by simulating the ventral and back channels in visual signal processing of the visual cortex of the brain. Dai et al. [4] discussed a parallel multilayer deep recognition architecture, which has stronger and more general feature extraction capabilities and thus conducts identification research on human behavior. Jaouedi et al. [5] established a human behavior detection and recognition model using the new single-lens multibox detector (SSD) algorithm to identify human behavior better from the monitoring video, and the model shows high precision and high speed rate. Xu and Qiu [6] proposed a deep time residual system for daily life activity recognition with team members. The deep time residual model of the human activity identification system was established, which improved the performance of the human identification system. Bakshi [7] proposed a new human activity recognition structure based on multisensor data. The wearable sensor human activity recognition based on the imaging time series was proposed. The image recognition was carried out by computer vision technology. The results showed that the system has better accuracy and F1 value. Tian et al. [8] proposed a new method (paired diversity measure and selective integrated learning based on the optimization of luminous worms to identify the human behavior) [8]. Data sets are collected from different parts of human body, including chest, waist, left wrist, left ankle, and right arm, to evaluate, which shows that the method has a high accuracy rate.

RETRACTED

Xie and Grossman [9] developed a CNN framework of crystal graph, which can learn the properties of materials directly from the connection of atoms in crystals. Finally, it shows how to use this information to discover the empirical rules of material design. Chen and Jahanshahi [10] proposed a deep learning framework based on CNN and Naive Bayes data fusion scheme (NB CNN), which is used to analyze a single video frame for crack detection of nuclear power plant components. Hatamzadeh et al. [11] put forward a robust and flexible neural network method based on a neural network to solve the background processing problem of difficult scenes and achieves better results. Ai et al. [12] built a toy model and simulated the model in the double *β*. The three-dimensional convolution and residual neural network are used in the charge track of the background. Through the test of the classification ability of the model, it is found that the three-dimensional structure and the overall depth of the neural network significantly improve the classification accuracy of the classifier. Under different conditions, the method is still stable and universal. Based on CNN, Hur et al. [13] proposed an efficient method for human activity identification, which accurately infers the correlation between the signal values of three-dimensional continuous sensors, and through experimental analysis, it is concluded that the accuracy of the method in the test data set is higher than other advanced methods. Ilyas et al. [14] proposed an improved MDK RESNET for CNN. The network extracts the characteristics between sampling points of different intervals, reduces the influence of environment background and camera shielding, and shows the effectiveness of the network in the results. Teng et al. [15] proposed a hierarchical CNN with local loss. It can realize human activity recognition using CNN based on local loss in ubiquitous and wearable computing. The results show that for the tested baseline architecture, local loss is better than global loss.

RETRACTED

In conclusion, the research on human activity recognition is abundant in the world, and there are many researches on the improvement and application of CNN. In addition, many researchers have applied a neural network to human activity recognition [16]. But most of the research knowledge simply carries on the identification analysis to the human daily activities, but in other fields such as sports the application is less. Therefore, this research will be based on CNN to identify and analyze the body behavior after the exercise training, so as to provide reasonable suggestions for the exercise training, and has certain guiding significance for the regulation of the intensity of sports training [17]. Finally, we can realize the reasonable training mode and improve the training level.

## 2. Detection of Body Behavior Characteristics after Sports Training Based on CNN

### 2.1. Construction of General Model of Body Characteristics of Athletes after Training

At present, there are many models for human behavior feature detection, such as SSD model proposed by some scholars to detect human behavior in subway and adaptive tracking frame scale adjustment model of particle space position proposed by some scholars to detect effective features. Although the feature detection models established by most scholars are of great practical value, it is undeniable that a large number of studies only focus on pedestrian movement detection, with less feedback on body information. Therefore, this study will combine the behavior detection model to analyze the body behavior of athletes after sports training according to the feedback information to improve the quality of sports training.

For the collection of body behavior characteristics after sports training, the target is extracted from the video sequence, that is to say, the body characteristics of athletes need to be obtained from the video image [18]. The body characteristics of athletes are mainly obtained from sports. In order to analyze the body characteristics scientifically and reasonably, firstly, the dynamic model of the body is analyzed, and the overall simplified model of the body characteristics is constructed, as shown in Figure 1.

RETRACTED

As shown in Figure 1, the human body changes from exercise training to rest state, and the most important change is the bone joint part supporting sagittal plane movement during the exercise. Figure 1 shows that the model of muscle body features mainly includes the lateral condyle of femur, medial condyle of femur, anterior cruciate ligament, posterior cruciate ligament, lateral meniscus, tibia, patellar ligament, and patellar joint surface in the skeleton. Firstly, the body characteristics of the exercise are studied. The changes of the body characteristics after training are analyzed [19]. The model is used to design the drive mode of the muscle body characteristics. The calculation method of the potential energy of the muscle feature movement is shown in the following equation:

(1) $$\begin{array}{c} P=\sum_{i=0}^{6}m_{i}gz_{i}, \end{array}$$

where *i* represents the number of rotational degrees of freedom in the model, *m* represents the mass of athletes, *g* is the acceleration of gravity, *g*=9.8(m/s)^2^, and *z* represents the longitudinal displacement caused by the rotation of the skeleton in the movement. At this time, in the motion image, we need to use visual technology to detect and analyze the motion end and joint points of the human body, and at the same time, it is necessary to recognize the motion of the human body in the video. In this study, according to the body feature model of human motion, the skeletal features of the human body during and after exercise are analyzed. The framework of 3D posture action recognition based on the human body is shown in Figure 2.

As shown in Figure 2, the framework is based on human behavior information. According to relevant research, the serialized spatial information can form human behavior information. Therefore, the skeleton sequence information of the human body is preprocessed as the data in video image recognition. The feature map of the body is processed into the original bone feature map and the moving skeleton feature map to fuse the features again, and the skeleton feature map is obtained by removing the redundant information, and finally, the 3D posture movement modeling and recognition of the human body can be realized. However, the limited number of human skeleton key points will also show the sparsity in the spatial dimension. It is unreasonable to extract information directly as a video sequence. Therefore, in order to encode effectively the limited skeletal action sequence information into rich two-dimensional spatial information, in this study, more effective information in the relative position coordinates between bones is considered. The left shoulder, right hip, and center hip are selected as reference points to calculate the relative sitting standard, as shown in the following equation:

(2) $$\begin{array}{c} V_{tk}≜\left\{X_{t}-r_{k}\right\}, \end{array}$$

where represents the set of bone points relative to the *k*th reference point at time *t*, *r*_*k*_ represents the space coordinates of the reference points of the *k*th reference point, and *X*_*t*_ represents the sequence value of bone points at time *t*. In addition, considering the external factors in the complex training environment, Savitzky–Golay smoothing filtering algorithm is used to filter the data and remove the noise in the data, as shown in the following equation:

(3) $$\begin{array}{c} X_{t}=\frac{\left(X_{t-2}+12X_{t-1}+17X_{t}-3X_{t+2}\right)}{35}, \end{array}$$

where *X* represents the spatial sequence. After filtering, the end and joint points of human motion are found, and the transfer function of the body mechanism is obtained, as shown in the following equation:

(4) $$\begin{array}{c} L=K-P. \end{array}$$

In addition to the determination of the transfer function, it is also necessary to obtain the mechanical equation under the driving mode of the body characteristics as follows:

(5) $$\begin{array}{c} \frac{\text{d}}{\text{d}t}\left[\frac{\partial L}{\partial {\dot{q}}_{i}}\right]-\psi_{0}\frac{\partial L}{\partial q_{i}}=\sigma_{\psi }T_{i},\;i=\left(1,2,\ldots ,6\right), \end{array}$$

where *L* is the transfer function of the equation, *ψ*_0_ is the variance matrix of the sampled data, and *σ*_*ψ*_ is the number of snapshots. The preprocessing work is to expand the bone points under each reference point into a one-dimensional vector and then superimpose multiple virtual vectors on the feature image to form a gray image in two-dimensional space. Finally, the gray images of all reference points are combined into three-dimensional space information. And according to the relevant research, the improvement of human action recognition results can be determined by the motion information obtained by bone dominant calculation. Therefore, the explicit calculation of bone motion information by equation (4) is as follows:

(6) $$\begin{array}{c} M_{t}=X_{t+1}-X_{t}, \end{array}$$

where *M*_*t*_ represents the motion information between adjacent frames and *X*_*t*_ represents the set of bone points obtained after preprocessing.

RETRACTED

### 2.2. Body Behavior Recognition Model after Sports Training Based on CNN

CNN was first used in two-dimensional image recognition, which is composed of five layers, including input layer, convolution layer, output layer, pooling layer, and fully connected layer. The input layer is the input signal, which is processed by the convolution layer and the pooling layer, and the target features in the image information are extracted layer by layer. The fully connected layer is used to classify the preprocessing information and finally output through the output layer. However, since this study is to extract the body behavior after human movement from the video, the ordinary two-dimensional image processing is obviously not good. Therefore, this study will use the three-dimensional convolution neural network model to extract the spatial information sequence in the video, and its structure diagram is shown in Figure 3.

Figure 3 shows that there are many sampling points in the input layer of the CNN model, which is conducive to extracting information from video from multiple angles and preserving the target features of video to the greatest extent. The convolution layer is the first hidden layer of the convolution neural network, different from the fully connected layer. The convolution layer and the input layer adopt local connections. Ten filters are selected to remove the noise of information. Ten different feature maps are obtained by the convolution layer. The pooling layer is the second hidden layer in the network, which is used to extract the characteristics of time. The whole connection layer is the third hidden layer in the network, which connects the pooling layer and the output layer and classifies the processed information by the output layer. The function of the output layer is to classify and output the final information. After continuous training in complex scenes, the human body needs to rest for a short or long time [20]. The recognition of body behavior characteristics after training is to recognize the fatigue degree of the human body after exercise. Therefore, four neurons were set in the output layer to judge the results according to the characteristics of the athletes' body behavior after training, which were extreme fatigue, severe fatigue, mild fatigue, and no fatigue. The convolution layer pseudocode description is shown in Figure 4.

Based on the convolution neural network, the human body movement is detected. In the study, the recognition and classification framework of human body behavior after exercise is constructed as shown in Figure 5.

Figure 5 shows that the human body behavior recognition combines the feature pyramid network that can improve the detection performance, and according to the particularity of the feature map, the sequence generation network is also used. Then, the region of interest alignment proposed by mask R-CNN is used to process candidate feature maps and finally transmitted to the fully connected layer to realize the detection and recognition of collective behavior features [21].

RETRACTED

The learning and training process of CNN directly determines the effect of the model in practical application. In this study, the design of CNN learning and training uses the backpropagation method. Firstly, the preprocessed training data is input into the model, and the activation value of the neuron is obtained by forward calculation. Then, the weights and bias gradients are calculated using the reverse error, and the original weights and bias gradients are adjusted using the obtained weights and bias gradients. The activation function of the CNN is constructed, as shown in the following equation:

(7) $$\begin{array}{c} y_{g}^{c}\left(m\right)=f\left(x_{g}^{c}\left(m\right)\right), \end{array}$$

where *c* is the number of layers of the network, *g* is the *g* th feature graph in the layer, *m* is the *m*th neuron of the feature graph, *y*_*g*_^*c*^(*m*) is the output data, and *x*_*g*_^*c*^(*m*) is the input data. The activation functions of the convolution layer and the pooling layer are set as follows:

(8) $$\begin{array}{c} f\left(x\right)=a\;\tanh\left(bx\right), \end{array}$$

where *a* and *b* are constant terms, with values of 1.7159 and 2/3, respectively. The Sigmoid function is selected as the activation function of the fully connected layer and the output layer, as shown in the following equation:

(9) $$\begin{array}{c} f\left(x\right)=\frac{1}{1+e^{-x}}, \end{array}$$

where *x* represents time. In the convolution neural network, the connection between each layer is data transfer. The specific transfer relationship can be briefly analyzed as follows: firstly, the data of the first layer is sampled, and the data of the first layer is convoluted by convolution kernel with appropriate size to get the characteristic graph of the convolution layer as follows:

(10) $$\begin{array}{c} y_{g}^{2}\left(m\right)=f\left(\sum_{1}^{i}Y_{i,m}\times k_{g}^{2}+b_{g}^{2}\left(m\right)\right), \end{array}$$

where *Y*_*i*,*m*_ is the sampling point, *k*_*g*_^2^ is convolution core, and *b*_*g*_^2^(*m*) is the offset of the network layer. The transfer mode from the convolution layer to the pooling layer is shown in the following equation:

(11) $$\begin{array}{c} y_{g}^{3}\left(m\right)=f\left(\sum_{1}^{n}y_{g}^{2}\left(\left(\left(m-1\right)\right)\times 10+n\right)\times k_{g}^{3}+b_{g}^{3}\left(m\right)\right), \end{array}$$

where *k*_*g*_^3^ represents the convolution kernel and *b*_*g*_^3^(*m*) is the offset of the network layer. The connection between the whole connection layer and the pooling layer is to connect all the neurons as follows:

(12) $$\begin{array}{c} y^{4}\left(m\right)=f\left(\sum_{1}^{i}\sum_{1}^{q}y_{i}^{3}\left(q\right)\omega_{i}^{4}\left(q\right)+b^{4}\left(m\right)\right), \end{array}$$

where *ω*_*i*_^4^(*q*) represents the weight of the pooling layer neurons connected to the fully connected layer neurons and *b*^4^(*m*) is the bias. For the connection between the fully connected layer and the output layer, the function is shown in the following equation:

(13) $$\begin{array}{c} y^{5}\left(m\right)=f\left(\sum_{1}^{i}y_{i}^{4}\left(i\right)\omega_{i}^{5}\left(i\right)+b^{5}\left(m\right)\right), \end{array}$$

where *ω*_*i*_^5^(*i*) represents the weight of connecting neurons in the connecting layer to neurons in the output layer and *b*^5^(*m*) is the bias. Secondly, it is necessary to initialize the weights and biases in the CNN in order to provide conditions for the training and learning of the network model. Then, the learning rates of the convolution layer and the pooling layer are set, as shown in the following equation:

(14) $$\begin{array}{c} \gamma =\frac{2\lambda }{N{\text{shared}}_{g}^{c}\sqrt{n{\left(c,g,i\right)}_{N\text{input}}}}, \end{array}$$

where *N*shared_*g*_^*c*^ represents the number of neurons with shared weights in the *g* characteristic graph of the *c* layer in the network and *n*(*c*, *g*, *i*)_*N*input_ represents the number of neurons connected by the *i*th neuron in the *g* characteristic graph of the upper layer and the *c* layer. Finally, the learning rate calculation formula between the fully connected layer and the output layer is set as follows:

(15) $$\begin{array}{c} \gamma =\frac{\lambda }{\sqrt{n{\left(c,g,i\right)}_{N\text{input}}}}, \end{array}$$

where *n*(*c*, *g*, *i*)_*N*input_ represents the number of neurons connected by the *i*th neuron in the *c* characteristic graph of the upper layer and the *g* layer. In this convolution neural network model, all the connection weights and offsets between each layer are set.

RETRACTED

## 3. Application Analysis of Monitoring Model for Body Behavior Characteristics

### 3.1. Performance Analysis of Body Behavior Feature Detection Model

The simulation experiment is carried out on the Windows system platform. Firstly, the three-dimensional modeling software SolidWorks is used to establish the human body motion model, and the driving data of each joint is saved as text data format. Then the body behavior recognition system is developed using Python 3.5 programming language. The data set used in the study is NTU RGB+D, which is the largest known human 3D skeleton action recognition data set [22]. The data set can provide additional information such as depth image and human contour. Ninety percent of the data set is used as the training set of the model and 10% as the model performance test set. The training results of the model in the experiment are shown in Figure 6.

As can be seen from Figure 6(a), with the increasing number of iterations, the accuracy of the CNN model is rising. When the number of iterations reaches 8, the rising speed of the accuracy of the model begins to slow down [23]. Until the number of iterations reaches 40, it begins to flatten, and the accuracy of the model has reached about 99%. As can be seen from Figure 6(b), the training time of the CNN model is 7.1 s, and the time of the trained model in the test set is 3.8 s. Generally speaking, the detection time of the model is short, although it does not show a very fast retrieval speed. According to the accuracy of model training, it is difficult to achieve fast retrieval speed while the model has high accuracy [24]. However, the detection time of the CNN model in the study is only 3.8 s, which also shows that the CNN model designed in this study has high performance. In addition, Figure 7 is the loss function curve of the model in training and testing.

As shown in Figure 7, the loss of the model in the training set and the test set decreases with the increase in the number of iterations. The model loss in training is small, and the initial value of loss in actual detection is large. It can be seen that when the number of iterations of the model is 30, the optimal solution of the model is obtained. In order to understand the overall advantages and disadvantages of the body behavior feature detection model, the more practical and effective detection algorithm BPNN [25] in recent years is collected and compared with the traditional detection algorithm. The error detection rate analysis results of the three algorithms are shown in Figure 8.

As can be seen from Figure 8, with the increase of image pixel value, the false detection rate of various algorithms will continue to decline. But it is not difficult to see that the detection rate of the traditional Bayesian algorithm is at a very poor level. When the image pixel is only 10, the error detection rate of the BPNN algorithm is far less than that of the traditional Bayesian algorithm. When the image pixel value is increasing, the error detection rate of the BPNN algorithm decreases significantly, and when the pixel value reaches 80, the error detection rate of the BPNN algorithm has dropped to 0.001. However, it is undeniable that the detection algorithm supported by CNN is obviously better than the other two algorithms. When the image pixel value is only 10, the false detection rate of the algorithm has dropped to below 0.005. Although with the continuous improvement of the image pixel value, the false detection rate of the CNN algorithm has a downward trend, which is not as obvious as that of the BPNN algorithm. However, the false detection rate of the CNN detection algorithm after the image pixel value reaches 80 has completely dropped to below 0.0005, and the false detection rate is almost zero. To sum up, the error detection rate of the CNN algorithm designed in this study is the lowest from beginning to end, which indicates that the CNN has better detection efficiency. In addition, the advantages and disadvantages of the CNN recognition and detection are analyzed by comparing the prediction performance of each model. The BPNN model and the model under the traditional Bayesian algorithm are also selected to compare with the CNN body behavior feature recognition model proposed in the study. The comparison results are shown in Figure 9.

RETRACTED

From Figure 9, it can be seen that the area of the target detection model under the three algorithms is more than 0.5, which indicates that the target detection model has better recognition performance. It is not difficult to see that the overall comprehensive recognition rate of CNN recognition and detection model reaches 91.67%. The overall recognition rates of BPNN and the traditional Bayesian algorithm model are 90.12% and 86.39%, respectively, which are significantly lower than the CNN identification and detection model. The reason for the above results is that the three-dimensional convolutional neural network proposed in this study analyzes the time series in the video sequence and also describes the spatial sequence, so the detected information is more clear. In conclusion, the convolutional neural network has good recognition performance.

### 3.2. Practical Analysis of Body Behavior Feature Detection Model

The body behavior feature detection model based on the convolution neural network model is tested in practical application. Four volunteers are recruited to carry out the final practical detection, and the detection performance is evaluated through subjective and objective aspects. Four volunteers were asked to conduct 0.5 hour, 1 hour, 1.5 hours, and 2 hours of exercise training in the training ground at the same time. After the exercise training, the training stopped. After each group of training, the rest returned to the normal state, and the next period of training was conducted at the same time. The body line feature detection model was used to identify the subjects' movements. The final recognition results are shown in Table 1.

RETRACTED

As shown in Table 1, the detection results of the body behavior feature detection model for four subjects under different training amounts are different, but it is not difficult to see that the detection accuracy of the body fatigue degree of the subjects under different training amounts is high. Finally, according to the results obtained by four subjects after receiving the detection of body behavior characteristics, according to their own active evaluation and analysis of whether the results are helpful for training, the total score is set as 10 points, and the results are shown in Figure 10.

It can be seen from Figure 10 that the four volunteers all gave a high evaluation on the model proposed in the experiment. Only volunteer no. 4 scored lower than 9 on the model. The reason may be that the volunteers had different feelings and tests on their own physical condition after training, but the volunteer still scored 8.9 on the model.

## 4. Conclusion

With the advent of the intelligent era, human action recognition has become a key research topic in the world. How to analyze accurately the characteristics of human behavior in a complex environment has become a problem to be solved. Therefore, based on convolution neural network, this study proposes a body behavior feature analysis model after human movement training, aiming to make use of the excellent feature analysis ability of convolution neural network to analyze the body of the athletes in the video after training, so as to make training plans for the future training. Through the training and learning of CNN and the comparative analysis with other algorithms, it is verified that CNN has better prediction performance, and the optimal model is selected in the training when the number of iterations are 30. After that, through the analysis of the body characteristics of the recruited volunteers after different training, we know that the detection model in the experiment has a high detection rate for different degrees of body fatigue and also shows a high evaluation in the subjective evaluation. To sum up, the analysis model of body behavior characteristics based on convolution neural network has a high detection rate, and the classification of fatigue degree after the analysis of human body characteristics also has a high accuracy rate, which has a good theoretical significance for the future sports training management and training mode optimization.

## Figures and Tables

**Figure 1:** General simplified model of human body characteristics.

**Figure 2:** A framework for human 3D pose recognition.

**Figure 3:** Three-dimensional CNN model.

RETRACTED

**Figure 4:** Convolution layer pseudocode.

**Figure 5:** Classification framework of human body behavior recognition.

**Figure 6:** Training results of the model: (a) CNN training result and (b) time.

**Figure 7:** The loss function curve of the model.

**Figure 8:** Comparison of false detection rate of three algorithms.

**Figure 9:** Model recognition performance comparison results.

**Figure 10:** Volunteer subjective evaluation results.

**Table 1:** Detection results of body behavior feature detection model application.

Fatigue level	Project	Volunteer 1	Volunteer 2	Volunteer 3	Volunteer 4
Relaxed	Accuracy	0.8756	0.8564	0.8725	0.8375
	Recall	0.8631	0.8731	0.8675	0.8562
	F-score	0.8697	0.8629	0.8743	0.8655

Moderate	Accuracy	0.8347	0.8851	0.8631	0.8954
	Recall	0.8531	0.8792	0.8413	0.8435
	F-score	0.8326	0.8811	0.8520	0.8943

Severe	Accuracy	0.8463	0.8639	0.8721	0.8647
	Recall	0.8631	0.8413	0.8952	0.8469
	F-score	0.8623	0.8234	0.8461	0.8454

Extreme	Accuracy	0.8643	0.8974	0.8746	0.8505
	Recall	0.8465	0.8746	0.8518	0.8635
	F-score	0.8461	0.8415	0.8484	0.8849

## Data Availability

The data used to support the findings of this study are available from the corresponding author upon request.
